# Superoxide-Dismutase Deficient Mutants in Common Beans (*Phaseolus vulgaris* L.): Genetic Control, Differential Expressions of Isozymes, and Sensitivity to Arsenic

**DOI:** 10.1155/2013/782450

**Published:** 2013-08-28

**Authors:** Dibyendu Talukdar, Tulika Talukdar

**Affiliations:** ^1^Department of Botany, RPM College, University of Calcutta, Uttarpara, West Bengal, Hooghly 712 258, India; ^2^Department of Botany, Krishnagar Govt. College, University of Kalyani, West Bengal, Krishnanagar 741101, India

## Abstract

Two common bean (*Phaseolus vulgaris* L.) mutants, *sodPv 1* and *sodPv 2*, exhibiting foliar superoxide dismutase (SOD) activity of only 25% and 40% of their mother control (MC) cv. VL 63 were isolated in EMS-mutagenized (0.15%, 8 h) M2 progeny. Native-PAGE analysis revealed occurrence of Mn SOD, Fe SOD, Cu/Zn SOD I and Cu/Zn SOD II isozymes in MC, while Fe SOD, and Mn SOD were not formed in *sodPv 1* and *sodPv 2* leaves, respectively. In-gel activity of individual isozymes differed significantly among the parents. SOD deficiency is inherited as recessive mutations, controlled by two different nonallelic loci. Gene expressions using qRT PCR confirmed higher expressions of Cu/Zn SOD transcripts in both mutants and the absence of Fe SOD in *sodPv 1* and Mn SOD in *sodPv 2*. In 50 *μ*M arsenic, Cu/Zn SODs genes were further upregulated but other isoforms downregulated in the two mutants, maintaining SOD activity in its control level. In an F_2_ double mutants of *sodPv 1* × *sodPv 2*, no Fe SOD, and Mn SOD expressions were detectable, while both Cu/Zn SODs are down-regulated and arsenic-induced leaf necrosis appeared. In contrast to both mutants, ROS-imaging study revealed overaccumulation of both superoxides and H_2_O_2_ in leaves of double mutant.

## 1. Introduction

Superoxide radicals are ubiquitously generated in many biological oxidations within all compartments of the cell. The toxicity of superoxide radicals has been attributed to their interaction with other cellular constituents, in particular with hydrogen peroxide [1]. Superoxide dismutases (SODs; EC 1.15.1.1) are a family of metalloenzymes that catalyze the disproportionation of superoxide radicals into H_2_O_2_ and O_2_ and constitute the first line of defense against the toxicity of superoxide radicals [1, 2]. Based on the metal cofactor used by the enzyme, SODs are classified into three groups as iron SOD (Fe SOD), manganese SOD (Mn SOD), and copper-zinc SODs (Cu/Zn SOD) [3]. SOD isozymes are located in different cellular compartments [3]. Fe SODs are located in the chloroplast, Mn SODs in the mitochondrion and the peroxisome, and Cu/Zn SODs in the chloroplast, the cytosol, and possibly the extracellular space. Cu/Zn SOD is normally quite stable, due in large part to copper and zinc binding and oxidation of an intramolecular disulfide [3]. Copper serves as the catalyst for superoxide disproportionation, whereas zinc and the disulfide participate in proper protein folding [3].

Arsenic (As) is a ubiquitous toxic metalloid without known biological functions in higher plants [4, 5]. In recent times, the impact of irrigation with high As contaminated groundwater on soil and crops has drawn huge attention due to transfer of As to the food chain via the groundwater-soil-plant system [6–8]. As can induce oxidative stress through generation of reactive oxygen species (ROS) [4, 5], and moderate accumulation of ROS significantly affects nuclear gene expression [9]. ROS sensors could be activated to induce signaling cascades that ultimately impinge on gene expression. Alternatively, components of signaling pathways could be directly oxidized by ROS. Finally, ROS might change gene expression by targeting and modifying the activity of transcription factors [9].

Mutational strategy provides a powerful tool to study the genetic, physiological, and molecular mechanisms of plants' response to abiotic stresses [10–12]. Among the edible legumes, this tool has been successfully used in *Pisum sativum* L. *Lens culinaris* Medik. and *Lathyrus sativus* L. to decipher metal tolerance and accumulation [10, 11], role of ascorbate and glutathione in redox balance and stress tolerance [12, 13], to ascertain genetic basis of flavonoid deficiency [14], to assess gene-dosage effect on antioxidant defense [15], and tolerance to salinity stress [16]. Among the enzymatic defense components in edible legumes, two mutants differing in catalase deficiency have recently been isolated and their genetic basis has been characterized in lentil [11]. The importance of SOD in ROS metabolism, maintenance of DNA integrity and life span has been nicely demonstrated by analysis of mutants in microbes and animals [17, 18]. In higher plants, importance of SOD has been studied in transgenic plants overexpressing SODs [19], which often produced inconclusive results [20]. The effects of Zn availability on SOD activity were studied in novel *raz *(*requires additional zinc*) mutant of *Medicago truncatula*, manifesting the importance of SOD mutant to study genetics of metal tolerance in plants [21]. The importance of Mn SOD in plant growth and Fe SOD isozymes in early chloroplast development has recently been elucidated in different *Arabidopsis* mutants [19, 20]. Using mutagenic primers in RT PCR, mutations were induced in Cu/Zn SOD genes and a thermostable SOD was engineered in higher plant *Potentilla atrosanguinea* [22].

*Phaseolus vulgaris* L. or common bean is a widely grown food legume and is rich in antioxidant flavonoids and proteins [23]. Like many other edible legumes, beans are highly sensitive to arsenate form of arsenic [23, 24] and showed severe perturbations in different morpho-physiological, micromorphological, and biochemical parameters under As exposure [25]. An earlier study revealed significant alterations in SOD activity in leaves of common beans subjected to As treatment [25], although genetic basis of SOD activity, roles of different isozymes, and their expression pattern were not known. Information about structural and functional aspects of SOD isozymes could benefit agricultural crop production through a better understanding of the genetic programs by which plants optimize photosynthetic activity in their green tissues during diverse types of stress conditions [3, 22, 25]. As part of a broad strategy to develop novel and desirable mutants for stress response in grain legumes, induced mutagenic technique has been adopted and progeny with variant phenotype was screened for antioxidant capacity. In the process, four plants exhibiting severe SOD deficiency in leaves were isolated at EMS-induced M_2_ generation and advanced to next generation to perform a detail study. The objective of the present study was framed to (1) measure the foliar SOD activity, (2) identify and analyze the in-gel activity of different SOD isozymes, (3) trace the inheritance of SOD deficiency in intercrossed population, (4) investigate the gene expression pattern of mRNA transcripts of different SOD isozymes, and (5) detect the ROS accumulation in leaves of mother variety, two mutant lines, and F_2_-segregating progeny under untreated and As (50 *μ*M)-treated conditions. 

## 2. Materials and Methods

### 2.1. Plant Materials

Fresh and healthy seeds of common bean legume (*Phaseolus vulgaris* L. cv. VL 63) presoaked with water (6 h) were treated with freshly prepared 0.15% aqueous solution of EMS (Sigma-Aldrich) for 8 h with intermediate shaking at 25 ± 2°C. M_1_ seeds were sown treatment wise in completely randomized block design as reported earlier [14, 26]. During screening of antioxidant activity of M_2_ plants in 2010, three variant plants showing abnormally low foliar activity of superoxide dismutase were detected. Seeds of these three variant plants (mean 120 seeds plant^−1^) were harvested, separately, and were sown in next season (2011) to raise M_3_ progeny. Leaf SOD activity of respective progeny plants (a total of 210 plants) was again confirmed at M_3_ generation, and based on this primary observation, the mutants were tentatively designated as *Phaseolus vulgaris SOD-deficient mutant*. As no phenotypic abnormalities were observed, the progeny plants derived from these three variant M_2_ plants were tested for SOD activity in completely separate sets. Further biochemical and molecular characterizations of SOD enzymes were performed on these progeny plants. 

### 2.2. Culture Conditions and As-Treatment Protocols

Fresh and healthy seeds of common bean legume (*Phaseolus vulgaris* L. cv. VL 63), mutant plants, and their intercrossed F_2_-progeny plants were surface sterilized with NaOCl (0.1%, w/v) and continuously washed under running tap water followed by distilled water. Seeds were allowed to germinate in the dark in two separate sets on moistened filter paper at 25°C. Germinated seedlings were randomly placed in polythene pots (10 plants pots^−1^) containing 300 mL of Hoagland's No 2 nutrient media and were allowed to grow for 7 d. The plants were, then, subjected to 50 *μ*M sodium arsenate (As, MW 312.01 g/mol; technical grade, purity 98.5%, Sigma-Aldrich) keeping untreated plant as control. Untreated mother variety and mutant plants were designated as mother control (MC) and mutant control (MuC), respectively. Control and treated plants were allowed to grow for another 7 d. Nutrient solution was refreshed every alternate day to prevent depletion of nutrients as well as As in the course of the plant's exposure to the metalloid. The experiment was carried out in a completely randomized block design with three replicates in an environmentally controlled growing chamber under a 14 h photoperiod, 28/18 (±2°C), relative humidity of 70 ± 2%, and a photon flux density of 100 *μ*mol m^−2^s^−1^. 

### 2.3. Determination of SOD Activity and Electrophoretic Analysis of SOD Isozymes

Fresh leaf tissue (250 mg) was homogenized in 1 mL of 50 mM potassium phosphate buffer (pH 7.8) containing 1 mM EDTA, 1 mM dithiothreitol, and 2% (w/v) polyvinyl pyrrolidone (PVP) using a chilled mortar and pestle kept in an ice bath. The homogenate was centrifuged at 15,000 g at 4°C for 30 min. Clear supernatant was used for enzyme assays. All operations were performed at 0–4°C. Soluble protein content was determined using BSA as a standard [27].

SOD (EC 1.15.1.1) activity was determined by nitro blue tetrazolium (NBT) photochemical assay, according to Beyer Jr. and Fridovich [28]. In this method, 1 ml of solution containing 50 mM K-phosphate buffer (pH 7.8), 9.9 mM L-methionine, 57 *μ*M NBT, and 0.025% triton-X-100 was added into small glass tubes, followed by 20 *μ*L of enzyme extract. Reaction was started by adding 10 *μ*L of riboflavin solution (0.044 mg mL^−1^), and the absorbance of solution was measured at 560 nm. SOD activity was expressed as U (unit) mg^−1^ protein. One unit of SOD was equal to that amount which causes a 50% decrease of SOD-inhibited NBT reduction. SOD isozymes were individualized by native PAGE on 10% acrylamide gels and were localized by a photochemical method [28]. Activity-staining gels were incubated for 30 min in 50 mM K-phosphate buffer at pH 7.5 containing 2 mM KCN or 5 mM H_2_O_2_ or 5 mM NaN_3_. Cu/Zn-SODs are inhibited by KCN and H_2_O_2_; Fe SODs are inactivated by H_2_O_2_ and NaN_3_ but resistant to KCN and Mn SODs are resistant to all three inhibitors. Quantification of the bands was performed using a Gel Doc system (Bio-Rad Laboratories, Chennai, TN, India) coupled with a high sensitive CCD camera. Band intensity was expressed as relative transmittance units. Based on the observed variations, isozyme bands were assigned to putative loci following the earlier adopted principles [29]. Only clearly visible bands were scored in the present study.

### 2.4. Genetic Control and Allelism Test of SOD-Deficient Mutations

Inheritance of mutations controlling SOD deficiency was traced in segregating populations of F_2_ generation derived from MC × mutants. For allelism test, intercrosses were made between mutants. Chi-square test was employed to test the goodness of fit between observed and expected values for all crosses. Zymograms of SOD isoforms of leaf F_1_ and F_2_ plants were analysed and compared with parents. 

### 2.5. RNA Isolation and Relative Gene Expression through Quantitative RT PCR

Gene expression levels of different SOD isozymes of MC, MuC, F_2_-segregating progenies, and As-treated plants of *Phaseolus vulgaris* (*PvSOD*) were analyzed by quantitative reverse transcription polymerase chain reaction (qRT-PCR) technique. Total RNA was isolated from the young leaves of 14d-old *Phaseolus* leaves (control and treated in separate sets of experiment) using the RNA isolation kit (Chromous Biotech, Bangalore, India) and treated with DNaseI (Chromous Biotech, Bangalore, India) at 37°C for 30 min. The quality of total RNA samples was determined spectrophotometrically (Systonic, Kolkata, India) and by 1% agarose gel electrophoresis with 500 bp DNA ladder. First-strand cDNA was synthesized from DNase-treated RNA with oligo-dT primer and with MmuLV reverse transcriptase enzyme kit (Chromous Biotech, Bangalore, India) following manufacturer's instructions. Quantitative RT PCR of first stand cDNA was run on ABI Step-One Real Time PCR machine. Amplification was done in a total reaction volume of 50 *μ*L, containing template (first strand cDNA) 2.0 *μ*L, forward primer 2.0 *μ*L, reverse primer 2.0 *μ*L, 2 X PCR SYBR green ready mixture (Fast Q-PCR Master Mix, Chromous Biotech, India, Cat no. QCR 05/QCR 06), 25.0 *μ*L, and DEPC water 19.0 uL. The SOD primers for four isozymes (Cu/Zn-SODs I and II, Fe SOD, and Mn SOD) of *PvSOD *(Table 1) were constructed by Primer Express software with the search of available GenBank/legume databases [30]. The qRT-PCR cycling stages consisted of initial denaturation at 94°C (3 min), followed by 35 cycles of 94°C (5 s), 62°C (10 s), 72°C (10 s), and a final extension stage at 72°C (2 min). A melting curve analysis was performed after every PCR reaction to confirm the accuracy of each amplified product. Samples for qRT PCR were run in five biological replicates and two technical replicates. DEPC water for the replacement of template was used as negative control. RT-PCR reaction mixtures were loaded onto 2% agarose gels in TAE buffer. A 100 bp DNA ladder was run on every gel. The mRNA levels were normalized against a common bean *ubiquitin* as the housekeeping gene and the relative (to control) expression of target genes was calculated as 2^−ΔΔCt^; Ct is cycle threshold, following Livak and Schmittgen [31]. 

### 2.6. Detection and Imaging of Superoxide and H_2_O_2_ Radicals by Confocal Laser Scanning Microscopy

Detection and imaging of superoxide radicals in leaf sections was carried out using the fluorescence probe dihydroethidium (DHE), following the earlier method [32]. Bean leaf segments of approximately 30 mm^2^ were incubated for 1 h at 25°C, in darkness, with 10 *μ*M DHE prepared in 5 mM Tris-HCl buffer at pH7.4, and samples were washed twice with the same buffer for 12 min each. After washing, leaf sections were embedded in a mixture of 15% acrylamide-bisacrylamide stock solution, and 100 mm thick sections, as indicated by the vibratome scale, were cut under 10 mM phosphate-buffered saline (PBS). Sections were then soaked in glycerol: PBS (containing azide) (1 : 1 v/v) and mounted in the same medium for examination with a (CLSM) system (Carl Zeiss, LSM 780, Bangalore, India) using standard filters and collection modalities for DHE green fluorescence (*λ* excitation 488 nm; *λ* emission 520 nm) and Chlorophyll autofluorescence (Chl a and b, *λ* excitation 429 and 450 nm, resp.; *λ* emission 650 and 670 nm, resp.) as blue. H_2_O_2_ was detected by incubation with 25 *μ*M 2′ 7′-dichloro fluorescein diacetate (DCF-DA) (excitation 485 nm, emission 530 nm) [32]. A preinfused leaf sections with 1 mM tetramethylpiperidinooxy (TMP), a scavenger of superoxide radicals, and 1 mM ascorbate, a scavenger of H_2_O_2_ served as negative controls. 

### 2.7. Statistical Analysis

The results presented were the mean values ± standard errors obtained from at least four replicates. Statistical significance of mean values between control and treated seedlings was determined by Students *t*-test (two tailed) using Microsoft Excel tool pack “data analysis” 2007. Multiple comparisons among treatments were performed by ANOVA using software SPSS v. 10.0 (SPS Inc., USA), and means were separated by Duncan's multiple range test. A probability of *P* < 0.05 was considered significant.

## 3. Results and Discussions

### 3.1. Foliar SOD Activity and In-Gel Activity of Isozymes in Control and As-Treated Leaves

In crude extracts of leaves under unstressed condition, measurable total SOD specific activity in MC plants was 40.8 (±3.9) U mg^−1^ protein. SOD activity in progeny mutant plants was only between 25% (10.2 ± 2.2 U mg^−1^ protein) and 45% (19.1 ± 2.9 U mg^−1^ protein) of MC plants, exhibiting severe deficiency of foliar SOD level in the mutant plants. Based on SOD activity level, mutant population could be clearly separated into two groups of progeny plants; one group of plants coming from two M_2_ parent (total three plants detected in M_2_ generation) showed mean SOD activity of only 25% of MC plants while the other group possessed SOD activity of only 45% of MC SOD level. All the mutant plants were phenotypically similar to MC plants (figure not shown). 

The analysis of SOD activity by native PAGE showed the presence of four isozymes in leaves of MC plants (Figure 1). Isozymes were identified with specific inhibitors (KCN and H_2_O_2_) as an Mn SOD, Fe SOD, and two Cu/Zn SODs (I and II), representing 45, 30, and 25% of the total SOD activity, respectively (Figure 2). The band showing resistance to inhibition by KCN, H_2_O_2_, and NaN_3_ was identified as Mn SOD (Figure 3), whereas band manifesting resistance to KCN but sensitive to H_2_O_2_ and NaN_3_ was detected as Fe SOD (Figure 3). The other two isozymes were sensitive to both KCN and H_2_O_2_ but resistant to NaN_3_. Therefore, they were assigned as Cu/Zn SODs (Figure 3) with the more anodal band was detected as Cu/Zn SOD II (Figure 1). The Cu/Zn SODs I and II were identified as faint bands in comparison with other isoforms of SOD in leaves, representing only 15% and 10% of total SOD activity, respectively (Figures 1–3). 

Different scenario was encountered in two groups of mutant plants. A total of three isozyme bands were clearly visualized in leaves of mutant plants (Figure 1). Band position and inhibitor studies in comparison with MC plants revealed complete absence of Fe SOD in the group showing only 25% SOD activity of MC plants, while there was no detectable Mn SOD band in other group, exhibiting 45% SOD activity of MC plants (Figures 1–3). Based on this observation, the former group of mutant plants was designated as *sodPv 1* (*superoxide dismutase deficient Phaseolus vulgaris mutant 1*) while the latter was described as *sodPv 2 *(*superoxide dismutase deficient Phaseolus vulgaris mutant 2*). In *sodPv 1* mutant, bands representing Mn SOD, Cu/Zn SOD I, and CU/ZnSOD II performed 60%, 25%, and 15% of the total SOD activity, respectively (Figure 2). On the other hand, in *sodPv 2* mutant plants, major share (65%) of SOD activity was carried out by Cu/Zn SODs (45% by Cu/Zn SOD I and 20% by Cu/Zn SOD II) while rest (35%) was contributed by Fe SOD (Figure 2). 

Under 50 *μ*M As exposure, foliar SOD activity in treated mother plants was increased over MC by about 3-fold (121.9 ± 5.7 U mg^−1^ protein), indicating generation of excess superoxide radicals due to As treatment, and it is in agreement with earlier reports on As-treated *P. vulgaris*, *P. aureus*, *Lathyrus sativus*, and *Trigonella foenum-graecum* [3, 7, 25, 33]. Besides As, heavy metal-dependent induction of SOD activity was also found in crops like *Pisum sativum* [32], *Lens culinaris* [34], *Helianthus annuus* [35], and *Coffea arabica* [36]. In the present case, the increased SOD activity in treated mother plants was accompanied with enhancement of band intensity of leaf Fe-SOD and Cu/Zn SODs (I and II) over that of MC (Figure 1), representing 38% and 52% of the total SOD activity (Figure 2). By contrast, band corresponding the expression of Mn SOD was faint (Figure 1), representing 10% of total SOD expression under As exposure (Figure 2). In the similar treatment protocol, measurable SOD level compared to MuC varied nonsignificantly (*P* > 0.05) in the As-treated mutants. In native PAGE gel, Cu/Zn SODs bands became intensified and thick in both mutants (representing nearly 83% of total SOD activity in *sodPv 1* and 90% of that in *sodPv 2* mutant), but bands representing Mn SOD (17% of total SOD) and Fe SOD (10% of total SOD) were visualized as very faint and thin in *sodPv 1* and *sodPv 2* mutants, respectively (Figures 1 and 2). 

### 3.2. Genetics of SOD Deficiency and Isozyme Pattern in Phaseolus Mutants

The two mutants exhibited phenotypes similar to MC. The MC plants as well as the two mutants were purely homozygous for SOD expression, as revealed by preliminary screening of their self-pollinated progeny (data not shown). Reciprocal crosses between *sodPv 1 *as well as *sodPv 2 *and MC yielded F_1_ plants with normal level of SOD activity (ranged 37.7–43.2 U mg^−1^ protein, mean 40.3 ± 5.9 U mg^−1^ protein). Segregation of normal and SOD-deficient plant type showed good fit [*χ* ^2^ = 0.43 at 1 df (degrees of freedom), *P* < 0.05] to 3 : 1 in F_2_, indicating recessive nature of mutant traits. In order to ascertain the allelic relationships of genes controlling SOD deficiency in *Phaseolus*, *sodPv 1 and sodPv 2* were reciprocally crossed. All the F_1_ plants exhibited normal SOD activity (37.9–42.8 U mg^−1^ protein, mean 41.1 ± 3.7 U mg^−1^ protein) and zymogram phenotype identical to MC (Figure 4). However, in F_2_, out of 480 plants screened, 270 plants possessed SOD activity (38.3–43.7 U mg^−1^ protein, mean 40.9 ± 4.9 U mg^−1^ protein) and isozyme patterns similar to MC, while rest of the plants (210) exhibited deficiency in SOD activity and altered zymogram pattern. A careful examination of these 210 plants revealed further segregation, of which 88 plants were identified exhibiting SOD activity (mean 10.8 ± 3.3 U mg^−1^ protein, 25.2% of MC) and isozyme pattern (Fe SOD absent) like *sodPv1*, 101 plants were detected manifesting SOD activity (18.3 ± 4.9 U mg^−1^ protein, 44.8% of MC) and isozyme pattern (Mn SOD absent) similar to *sodPv 2* mutant, and rest 21 plants were isolated with SOD activity of 12.5% (mean 5.1 ± 2.8 U mg^−1^ protein) of MC and occurrence of only Cu/Zn SOD I and II isozymes as faint bands (Figure 4). Inhibition study confirmed the presence of only Cu/Zn SODs isozymes, and no Fe SOD and Mn SOD bands could be visualized in these 21 plants (Figure 5(A)). The plants were self-fertile but carried distinct necrotic spots on pod wall (Figure 5(B)). Therefore, considering the whole F_2_ population of total 480 plants, the segregation was consistent [*χ* ^2^ = 4.09 at 3 df (degrees of freedom), *P* < 0.05] with 9 : 3 : 3 : 1 in F_2_. The results strongly suggested recessive nature of both mutations which was manifested in inheritance of zymogram pattern of respective parents and was controlled by interactions between two different nonallelic loci. The recessive nature of null mutations in SOD isozyme loci was also reported in sunflower, maize, soybean, and other plants [37–39]. Obviously, in the presence of dominant alleles of both loci (*SOD Pv1*-*SODPV2*-), SOD activity and zymograms of isozymes were normal in the present MC plants. Absence of dominant alleles in the loci (either in the form of *sodPv 1*-*SODPv 2*- or *SODPv 1-sodPv 2-*) led to origin of two SOD-deficient mutants, differing distinctly in total SOD activity level and isozyme banding pattern. In the last class of progeny plants, double mutant recessive to both loci (*sodPv 1 *and *sodPv 2*) resulted in extremely deficient SOD level accompanied with phenotypic anomalies. 

### 3.3. Gene Expression of SOD Isozymes under Un-Stressed and As-Treated Conditions

The expression patterns of the Cu/ZnSODs I and II, Mn SOD, and Fe SOD genes in leaves of *Phaseolus* seedlings and two mutant lines under unstressed, and As-treated conditions were investigated by qRT-PCR (Figure 2). Under unstressed condition, the mRNA transcripts of Mn SOD, Fe SOD, Cu/Zn SODs I, and Cu/znSOD II isoforms were amplified by PCR in MC (Table 1, Figure 6). The mRNA transcripts of Cu/Zn SODs were also detectable in both *sodPv 1* and *sodPv 2* mutants, but there were no detectable transcripts of Fe SOD in *sodPv 1* mutant and no Mn SOD in case of *sodPv 2* mutants (Figure 6). Besides Cu/Zn SODs I and II, genes encoding Mn SOD transcripts were expressed in *sodPv 1* while those of Fe SOD were detected in *sodPv 2* mutant leaves (Figure 6). Relative expression pattern (compared to respective gene of MC) indicated that genes encoding Mn SOD as well as Cu/Zn SODs I and II transcripts in *sodPv 1* exhibited significantly (*P* < 0.05) higher level than those of MC values (Figure 7). Higher transcript levels of Cu/Zn SODs and Fe SOD compared to MC were also deduced in *sodPv 2* mutant leaves (Figure 7). Between the two mutants, gene expression of Cu/Zn SODs transcripts was markedly higher in *sodPv 2* mutant (Figures 6 and 7). 

Dramatic changes in gene expression pattern of SOD isozymes were observed in leaves of mother variety exposed to 50 *μ*M As. In comparison with unstressed condition (MC), relative mRNA levels of Cu/Zn SODs, Mn SOD, and Fe SOD were increased by 2-fold, 1.5-fold, and 3-fold, respectively, in treated mother (Figures 6 and 7). The Results suggested upregulation of Cu/Zn SOD, Mn SOD, and Fe SOD genes in response to As treatment of mother variety. Compared to MC, total SOD-specific activity was markedly increased in As-treated mother variety. Certainly, enhanced activity of Cu/Zn SODs and Fe SOD isoforms mainly contributed to this rise which can be attributed to As-induced transcriptional upregulation of both Cu/Zn SOD and Fe SOD genes. However, the declining activity of Mn SOD isoform, as manifested in native gel, was not in harmony with enhanced level of its mRNA transcript, indicating possible regulation of this isozyme at posttranscriptional level. 

In As-treated *sodPv 1* and *sodPv 2* mutants, mRNA transcripts of Cu/Zn SODs as amplified in qRT-PCR (Figure 6) were increased by about 2-2.2-fold over their corresponding levels in untreated control (MuC) and >3.0-fold in relation to MC (Figure 7). By contrast, reduced level of mRNA transcripts was observed for Mn SOD in *sodPv 1* and for Fe SOD in *sodPv 2* mutant exposed to As treatment (Figures 6 and 7). The results indicated As-induced upregulation of Cu/Zn SODs genes in both mutants but concomitant down-regulation of Mn SOD in *sodPv 1* and Fe SOD in *sodPv 2* mutant. Overexpression of mRNA genes controlling Cu/Zn SODs led to higher activity of this isozyme in zymogram, which was manifested as increasing band intensity and thickness in native PAGE. Likewise, declining activity of Mn SOD in *sodPv 1* and Fe SOD in *sodPv 2* mutant exposed to 50 *μ*M As treatment was presumably due to down-regulation of their respective genes governing mRNA transcripts. The results indicated differential regulation of SOD isozymes in both mutants, subjected to As treatment, presumably, balancing SOD activity in MuC levels (25% in *sodPv 1* and 45% in *sodPv 2* of MC). Differential regulations of SOD isoforms were also reported in cadmium-treated pea, transgenic alfalfa, salinity-induced lentils, and in many other plants experiencing stresses [32, 40–42]. Since Mn SOD and Fe SOD are proved to be mitochondrial and plastidic isoforms, respectively, their down-regulation in the present mutants of common beans could have adverse effect on plant growth, as observed in *Nicotiana* seedlings [43] and in transgenic *Arabidopsis* [19]. Interestingly, no As-induced oxidative damage and consequent retardation of plant growth was visible in any part of the present mutants, despite down-regulation of MnSOD in *sodPv 1* and Fe SOD in *sodPv 2* mutant under As exposure. Obviously, upregulations of Cu/Zn SOD I and II mRNA gene counterbalanced down-regulation of other SOD isoforms in the mutant plants, and presumably, are holding the key in response of both mutants to high As exposure. Compared to chloroplast, the amount of ROS produced by mitochondria is rather minor [44] and chloroplasts bear a particular risk of oxygen toxicity because molecular O_2_ can be photoreduced from photosystem I (PSI) [44]. The Cu/Zn SODs are the most prolific SOD isozymes in chloroplast [3, 43, 44], and therefore their overexpression has immense significance in ROS metabolism and oxidative balance in leaves of present As-treated mother plants and mutant lines. However, to what extent this SOD expression is modulating antioxidant defense components of *Phaseolus* seedlings and mutants in response to As treatment; further study is needed to decipher it. 

### 3.4. Gene Expression of F_2_-Segregating Progeny Plants under Unstressed and As-Treated Conditions

Compared to their respective parent, there were no significant alterations in mRNA levels and morphology of F_2_-segregating progeny plants either under untreated or As-treated conditions (data not shown) except in the double mutant. Compared to *sodPv 1 *and *sodPv 2* single gene mutant phenotypes, relative expression of mRNA genes encoding Cu/Zn SODs I and II was significantly low in the double mutant plants under untreated condition (Figures 7 and 8(a)). Furthermore, no mRNA transcripts of Mn SOD and Fe SOD were detected. The results indicated origin of double knockout mutant for SOD deficiency in segregating mutant progeny of *Phaseolus*. Upon exposure of the mutant to 50 *μ*M As for 7 days in hydroponics, Cu/Zn SODs transcript level is reduced further (Figures 7 and 8), suggesting As-induced down-regulation of the gene. Declining level of mRNA transcripts and complete absence of Mn SOD and Fe SOD resulted in extreme reduction of foliar SOD activity in the mutant, which was manifested as thin faint bands in zymogram of Cu/Zn SODs (Figures 4 and 5(a)). The plants became more stunted, and severe necrotic spots were visible on trifoliate leaves and petioles under As exposure (Figure 8(b)). It is noteworthy that necrotic spots were visible in the pod walls of the mutant even under untreated condition, and thus appearance of new necrotic spots on photosynthetic part after As treatment indicated onset of As-induced oxidative damage, triggered by severe SOD-deficiency. The result strongly confirmed incorporation of both recessive mutations in the mutant, impeding normal SOD activity through knocking out of its Mn SOD and Fe SOD isozymes and down-regulating of Cu/Zn SODs. It now seems likely that two different recessive mutations at SOD loci of *Phaseolus* affected two different isoforms of the same enzyme, leading to origin of SOD deficiency with differential gene expression and isozyme banding patterns in two mutant lines. Remarkably enough, the Cu/Zn SODs were normal to over-expressed in the presence of either Mn SOD (*sodPv 1*) or Fe SOD (*sodPv 2*) but were downregulated when both isoforms were absent in the double mutant. The highly contrasting phenotypes as observed between two single mutants and double mutant derived from their inter-crossed progeny are unique. The outcome is not in accordance with earlier reports on *Arabidopsis* mutants, manifesting severe albino phenotypes in double knockout of two Fe SOD isoforms and severe sensitivity to oxidative stress in its two single mutant parents [20]. Among the legumes, similar phenomenon was observed in catalase-deficient mutants in lentil [11], dwarf mutations, and flavonoid-deficient mutants of grass pea [14, 45]. Certainly, the dominant alleles of both loci are complimenting with each other in the present case to give normal gene expression of all four isozymes while incorporation of both mutations in homozygous recessive forms resulted in absence of both Fe SOD and Mn SOD expressions in double mutant. The results also revealed inheritance of SOD deficiency as stable mutations, null for Fe SOD in *sodPv 1* and Mn SOD isozymes for *sodPv 2*, along with As tolerance in advanced generations.

### 3.5. ROS Imaging by CLSM

The remarkable tolerance of *sodPv 1* and *sodPv 2* mutants but sensitivity of their double mutants and mother plants to As treatment was strongly evidenced by ROS imaging study. Occurrence of superoxide radicals was analyzed by CLSM using the fluorescence probe DHE. In MC, no red fluorescence due to superoxide radicals was detected (Figure 9(A)). However, in leaves of As-treated mother plants and two mutants, the red fluorescence was detected in trifoliate leaves with more severe effects on mother plants. It was not so abundant and localized only in vascular tissue, especially in xylem, and in epidermis of mutant lines (Figure 9(B)). In leaves of As-treated mother plants, the red fluorescence was detected in high amount in and around vascular regions, sclerenchyma, mesophyll, and epidermis (Figures 9(C) and 9(E)). When the leaf sections were preincubated with 1 mM TMP (a superoxide scavenger), a significant reduction of the fluorescence was observed (Figure 9(D)), thus exhibiting the specificity of DHE for detection and imaging of superoxide radicals in bean leaves. For H_2_O_2_ imaging, crosssection of MC leaves incubated with DCF-DA exhibited a bright green florescence which was highly restricted to only xylem regions of vascular tissue and sclerenchyma (Figure 9(F)). In As-treated leaves of mother plant, the green florescence was enhanced markedly in vascular bundles, sclerenchyma, mesophyll regions, and in epidermis (Figure 9(G)). Under untreated condition, DCF-DA fluorescence was localized only in xylem of two mutant lines (Figure 9(H)). No significant change in green fluorescence was observed in As-treated mutants (figure not shown). By contrast, the double mutant exhibited both red and green fluorescences, abundantly distributed in vascular tissues, epidermis, and mesophyll regions (Figures 9(I) and 9(J)). Quite interestingly, DCF-DA fluorescence was also distinctly visualized in leaf epidermal hair of As-treated double mutant (Figure 9(J)), which was not noticed in any other cases. A preincubation with 1 mM ascorbate considerably tamed the florescence (Figure 9(K)). The analysis of superoxides and H_2_O_2_ in leaf sections by CLSM showed an enhanced generation of superoxide radicals and H_2_O_2_/other peroxide and their abundant localizations in mesophylls of treated mother plant and double mutant, exposed to As. Overproduction of superoxides and H_2_O_2_ due to toxic metals/metalloids was distinctly screened by CLSM study in pea, *Medicago sativa*, and *Lupinus luteus* roots [32, 46, 47]. The absence of both red and green fluorescences in mesophyll tissues of present MC and two mutants and their abundant occurrence even in overlapping conditions with tissue autofluorescence (blue) in some cases in As-treated leaves of mother variety and double mutant plants suggested that ROS production could be associated with chloroplasts in these genotypes. It was also indicative that, despite SOD-deficiency, both mutant lines contained superoxides and H_2_O_2_ levels in their photosynthetic part/s quite effectively under As treatment. By contrast, higher magnitude of ROS generation and their accumulation in leaves of treated mother variety and double mutant plants was evidenced by enhanced florescence. This suggested foot printing of As-induced ROS generation and consequent oxidative damage to photosynthetic parts of these plant types. 

## 4. Conclusions

For the first time, two SOD-deficient mutants were isolated in *P. vulgaris* by EMS-induced mutagenic technique. The two mutants manifested normal growth. Native PAGE analysis and mRNA gene expression analysis revealed complete absence of Fe SOD in *sodPv 1* and Mn SOD in *sodPv 2* mutant leaves, while Cu/Zn SODs I and II were differentially expressed. The mother plants possessed all four isozymes. Genetic analysis revealed inheritance of SOD deficiency as recessive mutations, controlled by two different nonallelic loci; the occurrence of both alleles in recessive forms led to origin of a double mutant in F_2_. Under 50 *μ*M arsenic (As) treatment for 7 days, Cu/Zn SOD isozymes were markedly up-regulated in the two mutants and mother variety. Measurable SOD activity in the two mutants, however, changed nonsignificantly as Mn SOD in *sodPv 1* and Fe SOD in *sodPv 2* were downregulated in response to As. This was consistent with isozyme banding pattern in native PAGE. The As-treated mutants showed normal growth, and no significant accumulation of ROS was observed in leaf as revealed by ROS-imaging study. In the double mutant, total absence of both Mn SOD and Fe SOD transcripts was accompanied with significant down-regulation of Cu/Zn SODs, resulting in ROS accumulation at high magnitude during As exposure and appearance of necrotic spots on photosynthetic organs. The isolation and genetic characterization of two SOD-deficient mutants, differing in SOD constituents and gene expressions, can be used as novel molecular tools to decipher deeper roles of SOD in abiotic stress tolerance of common beans. Furthermore, the origin of a double mutant is a unique phenomenon as the mutant in self-fertilisation and, thus, can be incorporated in different genetic backgrounds to reveal crosstalk between SOD and different antioxidant defense machinery of edible legumes. A genetic manipulation can, therefore, be facilitated in antioxidant defense components in favor of better crop growth and yield.

## Figures and Tables

**Figure 1:** Zymogram of four isozymes of superoxide dismutase (SOD) in leaves of *Phaseolus vulgaris* L. Cv. VL 63 (mother variety) and two SOD-deficient mutant lines, *sodPV 1*, and *sodPv 2* under untreated (control) and 50 *μ*M arsenic- (As-) treated conditions; lane 1: mother control, lane 2: *sodPv 1 *(untreated), lane 3: *sodPv 2* (untreated), lane 4: treated mother, lane 5: treated *sodPv 1* mutant, and lane 6: treated *sodPv 2* mutant.

**Figure 2:** Activity of individual isozymes of superoxide dismutase (SOD) in mother control (MC), two mutants, *sodPv 1* and *sodPv 2*, and 50 *μ*M arsenic- (As-) treated mother variety VL-63 and two mutant lines in *Phaseolus vulgaris* L. Band intensities were expressed as relative transmittance (T) units. The results are means ± SE of at least three replicates, and same letters (four different types to represent four isozymes) above error bars denote nonsignificant (*P* > 0.05) differences among means by Duncan's multiple range test.

**Figure 3:** Inhibition (KCN, H_2_O_2_, and NaN_3_) study and visualization of SOD isoforms in native PAGE of leaf extracts of *Phaseolus vulgaris* cv. VL 63 (mother variety) and two SOD-deficient mutant lines, *sodPv 1*, and *sodPv 2*; lane 1: mother control (no inhibitor), lane 2: mother variety (KCN), lane 3: *sodPv 1 *(KCN), lane 4: *sodPv 2 *(KCN), lane 5: mother variety (H_2_O_2_), lane 6: *sodPv 1 *(H_2_O_2_), lane 7: *sodPv 2 *(H_2_O_2_), lane 8: mother variety (NaN_3_), lane 9: *sodPv 1*, and lane 10: *sodPv 2*. Note that complete absence of band at lane 7; Mn SOD is absent in *sodPv 2* mutant, and Fe SOD and Cu/Zn SODs are inhibited by H_2_O_2_ treatment.

**Figure 4:** In-gel activity of SOD isozymes in F_2_-segregating progeny derived from *sodPv 1* × *sodPv 2* mutants in *Phaseolus vulgaris* L.; lane 1: F_1_ progeny, and lanes 2–10: F_2_ progeny of which lane 2 is normal plant (all four isozymes visualized), lanes 3 and 4: progeny with *sodPv 1* phenotype (Fe SOD absent), lanes 5 and 6: progeny with *sodPv 2* phenotype (Mn SOD absent), lanes 7–10: double mutant (both Mn SOD and Fe SOD absent).

**Figure 5:** (A) Inhibition study of SOD isozymes produced by double mutant obtained from crosses between *sodPv 1* and *sodPv 2* mutants of *Phaseolus vulgaris* L.; lane 1: mother control (no inhibitor), lanes 2 & 3: double mutants (no inhibitor), lane 4: double mutant (KCN), lane 5: double mutant (H_2_O_2_), and lanes 6 & 7: double mutants (NaN_3_). Note that both Cu/Zn SODs I and II were inhibited by KCN and H_2_O_2_ in lanes 4 and 5, while visualized as, and normal faint bands by NaN_3_ at lanes 6 & 7, (B) appearance of necrotic spots (→) on pod wall of double mutant.

**Figure 6:** Representative agarose gel (2%) electrophoresis shows the amplified product of mRNA expression of SOD isozymes in mother control (MC), two SOD-deficient mutants, *sodPv 1* and *sodPv 2* under untreated conditions, and arsenic (50 *μ*M sodium arsenate, As)-treated mother variety and two mutants; lane 1: Mn SOD, lane 2: Fe SOD, lane 3: Cu/Zn SOD I, lane 4: Cu/zn SOD II, lane 5: housekeeping gene, and lane 6–100 bp DNA ladder (bold white arrow 200 bp).

**Figure 7:** Relative expressions of genes governing mRNA transcripts of four SOD isoforms in leaves of mother control (MC) variety VL 63 of *Phaseolus vulgaris* L., two SOD-deficient mutants, *sodPv 1* and *sodPv 2*, and a double mutant (DM) type derived from F_2_ progeny of *sodPv 1* × *sodPv 2* mutants under untreated, and 50 *μ*M arsenic- (As-) treated conditions were quantified by quantitative reverse transcription-polymerase chain reaction (qRT-PCR). The mRNA levels were normalized with respect to housekeeping gene *ubiquitin *and are expressed relative to those of control (MC) value, which were arbitrarily given a value of 1. Data are means ± SE of five biological replicates and two technical replicates. Single asterisks denote upregulation (at least 2.0-fold), and double asterisks represent down-regulation (at least 2.0-fold) of genes with respect to control values.

**Figure 8:** (a) Representative agarose gel (2%) electrophoresis shows the amplified product of foliar mRNA expression of Cu/Zn SODs isozymes in mother control (MC, lanes 1, and 2) and a double mutant derived from *sodPv 1* × *sodPv 2* mutants under untreated (lanes 3 and 4) and arsenic (50 *μ*M sodium arsenate) treated (lanes 5 and 6) conditions, and (b) normal trifoliate leaflets (MC) and leaflets showing necrosis (→) in double mutant.

**Figure 9:** Representative imaging of superoxide radicals and H_2_O_2_ productions in *Phaseolus vulgaris* L. leaves by CLSM. Images are developed from several optical sections collected by confocal microscopy showing the autofluorescence (blue; excitation at 633 nm, emission at 680 nm) and fluorescence due to DHE and DCF-DA. A–E, (I) superoxide-dependent DHE fluorescence (red) in leaf cross sections from mother control (A) and arsenic (As)-treated (B–K) leaves; (B) As-treated *sodPv 1* mutant, (C) As-treated mother plants, (D) for the negative control, leaves were incubated with 1 mm TMP, a superoxide scavenger, (E) magnified view of leaf mesophyll with red fluorescence and autofluorescence, (I) red fluorescence in leaf section of double mutant, F–H, J, and (K) H_2_O_2_-dependent DCF-DA fluorescence (green) in leaf cross sections; (F) MC leaves, (G) As-treated mother plants, (H) As-treated *sodPv 2* mutant, (J) green fluorescence in leaf tissues along with epidermal hair of double mutant, (K) as a negative control, and leaves were incubated with 1 mm ascorbate (ASC), which acts as a H_2_O_2_ scavenger. The results are representative of at least three independent experiments. Ep: Epidermis; Hr: hair; Ms: mesophyll cells; Scl: sclerenchyma; Xyl: xylem vessels. Bars = 50 *μ*m.

**Table 1:** Oligonucleotides used for qRT-PCR analysis of target gene expressions of superoxide dismutase (SOD) isozymes in *Phaseolus vulgaris* L. mother cv. VL 63 and two of its SOD-deficient mutant lines. F1—forward primers and R1—reverse primers.

Target genes	Oligonucleotide sequence (5′→3′)	Amplicon size (bp)
Mn SOD	F1-AGTCAAGTTGCAGAGTGCAATCAAGTTC-	143
	R1-CAAAGTGATTGTCAATAGCCCAACCTAAAG-	
Fe SOD	F1-AACAAGCAAATAGCCGGAACAGAACTAAC-	127
	R1-AGAAATCGTGATTCCAGACCTGAGCAG-	
Cu/Zn SOD I	F1-GGCTGTATGTCAACTGGACCTCATTTCA-	139
	R1-TGTCAACAATGTTGATAGCAGCGGTG-	
Cu/Zn SOD II	F1-GGATATATGGCATCTGTAACTCATATGC-	115
	R1-GCATAAGAATGCTGATAGACAGGGTC-	
*Ubiquitin* (housekeeping gene)	F1-GCTCTCCATTTGCTCCCTGTT-	144
	R1-TGAGCAATTTCAGGCACCAA-	
